The article "Controlled Decompression Alleviates Brain Injury via Attenuating Oxidative Damage and Neuroinflammation in Acute Intracranial Hypertension" was retracted in 2023. Reasons: signs of a paper mill; compromised peer review; unreliable results or conclusions.

# Controlled Decompression Alleviates Brain Injury via Attenuating Oxidative Damage and Neuroinflammation in Acute Intracranial Hypertension

**DOI:** 10.1155/2022/1936691

**Published:** 2022-02-09

**Authors:** Chonghui Zhang, Xiao Qian, Jie Zheng, Pu Ai, Xinyi Cao, Xiaofei Pan, Tao Chen, Yuhai Wang

**Affiliations:** Department of Neurosurgery, The 904th Hospital of PLA, Medical School of Anhui Medical University, Wuxi, Jiangsu 214044, China

## Abstract

**Background:**

The benefits of controlled decompression (CDC) for patients with acute intracranial hypertension especially in terms of alleviating the complications caused by rapid decompression (RDC) have been confirmed by clinical studies. This study is aimed at evaluating the therapeutic potency of CDC with ubiquitin C-terminal hydrolase-L1 (UCH-L1) and glial fibrillary acidic protein (GFAP) by investigating the potential molecular mechanism in the acute intracranial hypertension (AICH) rabbit model.

**Methods:**

Male New Zealand white rabbits were randomly subdivided into the sham-operated (SH) group, CDC group, and RDC group. Blood plasma samples and brain tissue were collected 2 days before operation (baseline) and at 3, 6, 24, and 72 hours after operation to measure the levels of UCH-L1, GFAP, oxidative stress indicators, and inflammatory cytokines by performing ELISA or Western blot. The neurological score of the rabbits and brain water content was graded 24 h after surgery. qPCR, immunofluorescence, and FJ-C staining were conducted.

**Results:**

CDC improved neurological function, lowered brain water content, ameliorated neuronal degeneration, attenuated oxidative damage, and inflammatory responses to a greater extent than RDC. Plasma UCH-L1 level was significantly lower in the CDC group at 3 h postoperatively than in the RDC group. CDC reduced plasma GFAP levels to various degrees at 3 h, 6 h, and 24 h postoperatively compared with RDC. Immunofluorescence confirmed that the expression of UCH-L1 and GFAP in the cortex of the CDC group was lower than that of the RDC group.

**Conclusions:**

Our data collectively demonstrate that CDC could attenuate oxidative damage and inflammatory responses, downregulate UCH-L1 and GFAP levels, and contribute to an improved neuroprotective effect compared with RDC.

## 1. Introduction

Acute intracranial hypertension (AICH) is one of the most common causes for death and disability of patients suffering from traumatic brain injury (TBI) and hypertensive cerebral hemorrhage. The persistent high cranial pressure has been reported to be associated with poor prognosis and especially high mortality in adults with severe TBI [1, 2].

Decompressive craniectomy is constantly applied in the intervention of AICH [3, 4]. Unfortunately, in the wake of the rapid release of intracranial pressure, decompressive craniectomy may bring about unfavorable complications, such as acute intraoperative encephalocele, delayed hematoma, consequently contributing to the already dismal prognosis, and high mortality and disability rates. Meanwhile, the effect of decompressive craniectomy on improving the long-term prognosis of patients remains questionable in the medical community [5]. In contrast to the conventional surgery of decompressive craniectomy, controlled decompression (CDC) features a slow and gradual release of intracranial pressure under the parameters of ICP monitoring. A prospective randomized controlled cohort trial confirmed that CDC could reduce the 30-day all-cause mortality rate and improve the 6-month GOS-E scores of patients. In addition, CDC was proved to be more effective in reducing the incidence of intraoperative brain swelling, delayed hematoma, and posttraumatic cerebral infarction in patients compared with rapid decompression (RDC) [6]. Nevertheless, the potential molecular mechanisms and therapeutic effect of CDC warrant further analysis in the laboratory.

The article "Controlled Decompression Alleviates Brain Injury via Attenuating Oxidative Damage and Neuroinflammation in Acute Intracranial Hypertension" was retracted in 2023. Reasons: signs of a paper mill; compromised peer review; unreliable results or conclusions.

Recent clinical trials have explored the reliability and accuracy of various brain-specific biomarkers as indicators of TBI progression and prognosis [7, 8]. As the most promising candidate biomarkers, UCH-L1 and GFAP as tandem have recently been approved by the US Food and Drug Administration (FDA) for the assessment of intracranial injury in patients with TBI [9]. UCH-L1 is a cytoplasmic dedifferentiating enzyme specifically expressed in neurons and accounts for 1-5% of total proteins in the brain. As an integral component of the axonal skeleton, UCH-L1 plays a key role in axonal transport [10]. GFAP is a monomer of intermediate filament protein, a major component of the astrocyte skeleton, and a highly specific biomarker of the central nervous system (CNS). GFAP functions to maintain the cytoskeletal structure of glial cells and to bolster mechanical strength [11]. The aberrant expression of UCH-L1 and GFAP could indicate the severity of TBI from the perspective of neurons and astrocytes, respectively. A plethora of studies have applied animal models of TBI and cohorts of patients and reported that the elevated levels of plasma UCH-L1 and GFAP indicate the severity of the injury and the prognosis of patients, thereby substantiating UCH-L1 and GFAP as the ideal biomarkers in clinical practice [12, 13].

The objective of the current study is to verify the neuroprotective effect of CDC in the AICH model of rabbits by analyzing the levels of UCH-L1 and GFAP and to explore whether CDC alleviates brain injury via attenuating oxidative damage and neuroinflammation.

The article "Controlled Decompression Alleviates Brain Injury via Attenuating Oxidative Damage and Neuroinflammation in Acute Intracranial Hypertension" was retracted in 2023. Reasons: signs of a paper mill; compromised peer review; unreliable results or conclusions.

## 2. Material and Methods

### 2.1. Animals

Male New Zealand White rabbits (body weight = 2000 to 2500 g) were enrolled in the current study. The rabbits were raised under standard laboratory condition with a 12 h light/dark cycle at the controlled temperature of 22°C and humidity of 50%. The animals were granted free access to water and fodder 12 hours before the surgery. All the experimental procedures were carried out between 9:00 AM and 5:00 PM. The design and protocol of the current study were approved by the Ethics Committee of Wuxi Clinical College of Anhui Medical University (Hefei, Anhui Province, China); the experiments were performed in accordance with the Guide for the Care and Use of Laboratory Animals prescribed by the National Institute of Health. Every effort has been made to diminish the suffering of the animals during the experiment.

### 2.2. Experimental Design

Rabbits were randomly divided into three groups, including the SH group (*n* = 30), CDC group (*n* = 30), and RDC group (*n* = 30). The rabbits were anesthetized by intravenous injection of 3% pentobarbital (dose = 30 mg/kg). The dose would be increased if necessary. The rabbits were fixed in a prone position on a platform, their heads were disinfected with 75% alcohol, and local anesthesia was applied by using 0.5 mL of lidocaine. All surgeries were performed by the same surgeon. The vital signs of the rabbits were expected to remain principally stable during the surgery, and the temperature was maintained at 37°C by using a thermostatic blanket. After the procedure of anesthesia was completed, the scalp of the rabbit was incised longitudinally along the midline. A dental drill (JSDA, cat#JD700, China) was used to drill two holes (diameter = 0.5 cm) at a distance of 0.5 cm from the sagittal suture and coronal suture on the left and the right side. The structure of the dura was maintained intact during the drilling. A latex balloon was attached to an anesthesia epidural catheter (10 cm in length and 1 mm in diameter), was used to pierce through the bony hole towards the frontotemporal lobe, and was connected to an external pressure pump. Afterward, the ICP sensor (Codman, Johnson and Johnson Medical, cat#82-6635, USA) was vertically inserted into the brain tissue at a depth of 1 cm through the right bone hole. Dental cement (Dentsply, Jeltrate Alginate Impression Material, USA) was used to seal the two bone holes.

In the RDC group and the CDC group, normal saline (NS) was injected into the balloon via the pressure pump to increase the intracranial pressure to the extent of 38 mmHg and was maintained for 30 min. The fluid was rapidly withdrawn from the balloon in the RDC group, yet was slowly released from the balloon in the CDC group for 30 min. In the SH group, the epidural balloon was placed without the injection of NS, and then, the balloon was removed 30 min later. The experiment would be suspended immediately in the event of dilated pupil at the ipsilateral side of injury, deep and slow breath, and slowed heart rate. When the experiment approached the end, the epidural balloon and ICP probe were removed, the bone foramen was resealed, and the scalp incision was sutured. After the animals were resuscitated from the surgery, they were sent back to the animal house and were fed ad libitum.

The article "Controlled Decompression Alleviates Brain Injury via Attenuating Oxidative Damage and Neuroinflammation in Acute Intracranial Hypertension" was retracted in 2023. Reasons: signs of a paper mill; compromised peer review; unreliable results or conclusions.

### 2.3. Neurological Function Scoring

24 hours later, the neurological function scores of rabbits were independently observed and recorded by a researcher who was blind to the purpose and design of the experiment. The scoring system covers the aspects of Appetite, Activity, and Deficits, each of which ranged on a scale from 0 to 6. A higher score represents improved neurological function and vice versa. The detailed scoring standard refers to previous studies by Chen et al. [14].

### 2.4. Brain Water Content

Brain water content was evaluated by using the wet and dry weight method. Flesh brain tissue from compressed hemispheres in three groups of rabbits was harvested. The wet weight was precisely measured by an electronic balance (±0.01 mg). The dry weight was weighed after the brain tissue was dried in an oven at 100°C for 24 h. The following formula was used to assess the brain water content: brain water content (%) = (wet weight − dry weight)/wet weight × 100%.

### 2.5. Collection of Plasma and Brain Tissue Specimen

Plasma and brain tissue samples were collected from 6 rabbits in each group at 2 h preoperatively and at 3 h, 6 h, 24 h, and 72 h postoperatively. The rabbits were anesthetized using 3% pentobarbital (dose = 30 mg/kg) and were placed in the supine position. Intravenous hemostatic was used to pierce vertically into the heart. The blood that flowed into the tube with heparin anticoagulants was collected and was then centrifuged at 3000 g for 15 min at 4°C. The supernatant was extracted and immediately frozen on dry ice and was then stored at -80°C for the subsequent assay.

After the collection of plasma specimen, the thoracic abdomen of the anesthetized animal was cut open immediately, and the right auricle was snipped. After 500 mL of 0.1 M PBS was injected rapidly into the cardiac apex, 1000 mL of 4% paraformaldehyde (PFA) was injected rapidly, and the procedure was gradually slowed down to last 1.5 h in total. After the perfusion, the brain of the rabbits was collected and was prefixed using 4% PFA at 4°C for 24 h and was dehydrated at 4°C by using 30% sucrose solution until the brain shrank. The brain tissue sized approximately 8 mm × 5 mm × 5 mm was collected from the surrounding compressed area and was frozen on powdered dry ice.

The article "Controlled Decompression Alleviates Brain Injury via Attenuating Oxidative Damage and Neuroinflammation in Acute Intracranial Hypertension" was retracted in 2023. Reasons: signs of a paper mill; compromised peer review; unreliable results or conclusions.

### 2.6. Enzyme Linked Immunosorbent Assay (ELISA)

The levels of UCH-L1, GFAP, malondialdehyde (MDA), 8-iso-prostaglandin F2*α* (8-iso-PGF2*α*), tumor necrosis factor- (TNF-) *α*, interleukin- (IL-) 1*β*, IL-6, and IL-8 were measured by using commercialized ELISA kits (Nanjing Jiancheng, Bioengineering Institute, Nanjing, China), abiding by the manufacturer's instructions. The OD value of the well added with the diluted buffer was used as the baseline. Each well was measured sequentially, and an average value of the replicate wells was calculated based on the OD values of the plasma samples.

### 2.7. Western Blotting

Total protein was extracted from homogenized brain tissue samples by using RIAP lysis buffer (Beyotime; Nanjing, China). The loaded lysates in each lane were separated by using 12% SDS-PAGE. The proteins were transferred onto PVDF membranes (Millipore; USA), which were then blocked by using 5% nonfat dry milk. The membranes were incubated along with the primary antibodies overnight at 4°C. Subsequently, the membrane was washed three times using TBST and was then incubated with HRP-conjugated secondary antibody for 2 h at RT. Finally, the band of interested protein was revealed using a Bio-Rad imaging system (Bio-Rad, Hercules, CA, USA), and the signal intensity was quantified using the ImageJ software.

### 2.8. Real-Time Quantitative Polymerase Chain Reaction (qPCR)

The brain tissue in the vicinity of the injured area was lysed using Trizol reagent (Invitrogen; C.A., USA), following the instruction of the manufacturer. RT-qPCR was performed using SYBR Green Master Mix (Vazyme Biotech; Nanjing, China), and the primers were designed to amplify the products of qPCR. △Ct value of the target gene in each sample was obtained by subtracting the Ct value of GAPDH from the corresponding Ct value of each sample. The relative expression of each gene was determined by applying the classic 2^-△△Ct^ method was normalized to the level of GAPDH, which was employed as the housekeeping gene.

### 2.9. Fluoro-Jade C (FJ-C) Staining

FJ-C staining was conducted on the tissue sections following the method described by Schmued et al. [15]. The sections were mounted on the gelatin-coated slides, dried on a hot plate at 55°, immersed in alkaline ethanol solution for 5 min, and then washed twice using 70% ethanol. The slides were incubated in 0.06% KMnO_4_ (potassium permanganate) for 20 min on a shaker. The slides were then incubated in FJ-C solution on a shaker for 30 min in the dark, washed by double distilled water, air-dried, and sealed by using DPX (Cat# 44581, Sigma-Aldrich). FJ-carbon-labeled cells were visualized using a FITC-filter (excitation/emission ¼ 490/525 nm), and the number of FJ-C-positive neurons on the sections was counted under a microscope. All the images were saved as Tiff format.

The article "Controlled Decompression Alleviates Brain Injury via Attenuating Oxidative Damage and Neuroinflammation in Acute Intracranial Hypertension" was retracted in 2023. Reasons: signs of a paper mill; compromised peer review; unreliable results or conclusions.

### 2.10. Immunofluorescence

The collected brain tissue sections were washed three times using PBS for 15 min and were incubated in PBS for 15 min. The sections were blocked using goat plasma at 37° for 15 min. Subsequently, the slides were incubated overnight with primary antibodies against UCH-L1 and GFAP. After being washed by PBS in triplicate for 15 min in total, the slides were incubated with secondary antibody (Bioss, China) for 20 min and were washed by using PBS. After that, DAPI (Sigma-Aldrich) staining was performed. The slides were photographed using a confocal scanning microscope (Leica, Wetzlar, Germany) installed with the ImageJ software.

### 2.11. Statistical Analysis

Otherwise specified, the data in the current study were presented in the form of mean ± SEM. One-way ANOVA was used for multiple group comparison, followed by Bonferroni posttest or unpaired *t*-test on SPSS 20.0 (IBM, Chicago, USA) and GraphPad Prism 8.0 (San Diego, USA). A *P* value less than 0.05 indicates a statistically significant difference.

## 3. Results

### 3.1. Controlled Decompression Improved Neurological Function, Lowered Brain Water Content, and Attenuated Neuronal Degeneration

Neurological function scores and brain water content were measured at 24 h postsurgery to evaluate and compare the cerebral protective effect of the two surgical approaches. CDC, but not RDC, significantly improved neurological function scores (Figure 1(a)) and lowered brain water content (Figure 1(b)) in rabbits after AICH (*P* < 0.05). FJ-C staining was conducted 24 hours after the surgery to observe the extent of neuronal degeneration; the degenerated neurons would exhibit high intensity of fluorescence. Apparently, in spite of the high prevalence of degenerated neurons in both two groups (Figure 1(c)), the percentage of degenerated neurons in the CDC group was significantly downregulated than that in the RDC group (*P* < 0.001). The percentage of degenerated neurons was negligible in the SH group. Our data confirmed that CDC resulted in notably superior neuroprotective effect in the rabbits.

### 3.2. Controlled Decompression Attenuated Oxidative Damage

Oxidative damage was assessed by measuring the MDA, 8-iso-PGF2*α*, and SOD levels in the plasma and the cortex. After operation for AICH, the levels of MDA and 8-iso-PGF2*α* in plasma were increased at different degrees, while the levels of SOD were decreased. In the CDC group, the MDA and 8-iso-PGF2*α* levels were significantly lower at 6, 24, and 72 h after the operation when compared to the time-matched RDC group. On the contrary, the SOD levels were significantly higher at 24 and 72 h in the CDC group than in the RDC group (Figures 2(a)–2(c)). In addition, in the rabbit cortex of the CDC group, MDA and 8-iso-PGF2*α* were significantly lower than those in the RDC group, while SOD was significantly higher than those in the RDC group (Figures 2(d)–2(f)).

The article "Controlled Decompression Alleviates Brain Injury via Attenuating Oxidative Damage and Neuroinflammation in Acute Intracranial Hypertension" was retracted in 2023. Reasons: signs of a paper mill; compromised peer review; unreliable results or conclusions.

### 3.3. Controlled Decompression Attenuated Neuroinflammation

The inflammatory responses were evaluated for plasma TNF-*α*, IL-1*β*, IL-6, and IL-8 at 24 h after operation. qPCR results showed a higher expression of TNF-*α* (Figure 3(a)), IL-1*β* (Figure 3(b)), IL-6 (Figure 3(c)), and IL-8 (Figure 3(d)) mRNA in the RDC group compared with the CDC group. Similarly, plasma levels of the TNF-*α* (Figure 3(e)), IL-1*β* (Figure 3(f)), IL-6 (Figure 3(g)), and IL-8 (Figure 3(h)) were significantly increased after AICH. However, CDC significantly reduced the levels of above four inflammatory cytokines in plasma compared with RDC. The results suggest that AICH can lead to the increase of inflammatory cytokines in the plasma, which can be significantly attenuated by CDC.

### 3.4. Controlled Decompression Downregulated UCH-L1 and GFAP Expression in the Cortex of the Rabbits Postoperatively

To further explore the expression of the brain-specific biomarkers in the cerebral cortex of the rabbits, we detected UCH-L1 and GFAP at the compressed area of the cortex by conducting an immunofluorescence (IF) assay. The results showed that UCH-L1 was uniformly distributed and was weakly stained in the sham group, yet was strongly stained with coarse granules in the CDC and RDC group. The count of UCH-L1-positive cells in the CDC group was significantly less than that in the RDC group (*P* < 0.001) (Figure 4(a)). A small number of lightly stained GFAP-positive astrocytes were scattered in the SH group. In contrast, strong staining could be observed in the CDC and RDC groups. Intriguingly, the number of GFAP-positive cells in the CDC group was significantly less than that in the RDC group (*P* < 0.01) (Figure 3(b)).

### 3.5. Controlled Decompression Downregulated UCH-L1 and GFAP mRNA Levels in Rabbit Cerebral Cortex

In comparison with those in the SH group, UCH-L1 and GFAP mRNA levels in CDC and RDC groups were elevated to various degrees after AICH. UCH-L1 mRNA expression in the CDC group was significantly lower than that in the RDC group at 3 h postoperatively (*P* < 0.001) and at 6 h postoperatively (*P* < 0.01) (Figure 5(a)). GFAP mRNA in the CDC group was significantly lower than that in the RDC group at 3 h, 6 h, and 24 h postoperatively (*P* < 0.01) (Figure 5(b)). In summary, CDC reduces time-matched UCH-L1 and GFAP mRNA expression compared with RDC.

The article "Controlled Decompression Alleviates Brain Injury via Attenuating Oxidative Damage and Neuroinflammation in Acute Intracranial Hypertension" was retracted in 2023. Reasons: signs of a paper mill; compromised peer review; unreliable results or conclusions.

### 3.6. Controlled Decompression Downregulated UCH-L1 and GFAP Levels in the Plasma of Rabbits Postoperatively

We performed ELISA to reveal the changing patterns of UCH-L1 and GFAP levels in plasma in three groups. As illustrated in Figure 6(a), the plasma level of UCH-L1 peaked in the CDC group and RDC group at 3 h postsurgery and then decreased rapidly to approach the baseline values at 6 h postsurgery. Plasma UCH-L1 level in the CDC group was significantly reduced than that in the RDC group at 3 h postoperatively (*P* < 0.001). Nevertheless, the difference in plasma UCH-L1 between the two groups at 6 h postoperatively was not large enough to reach the extent of statistical significance. The aberrant elevation of plasma GFAP level persisted longer than that of UCH-L1. Of note, plasma GFAP level started to rise within 3 h postoperatively in the CDC group and RDC group, peaked at 6 h postoperatively, and plateaued above the baseline values until 72 h later (Figure 6(b)). Plasma GFAP expression at 3 h and 6 h postoperatively in the CDC group was lower than that in the RDC group (*P* < 0.001). Western blot shows that plasma expression of UCH-L1 and GFAP level at 3 h postoperatively was significantly lower in the CDC group, as opposed to that in the RDC group (*P* < 0.001) (Figure 6(c)).

## 4. Discussion

In the present study, we evaluate the neuroprotective effects of CDC and RDC by UCH-L1 and GFAP expression in plasma and cortex. The results concurred that CDC improved neurological function, lowered brain water content, and attenuated oxidative damage and inflammatory responses than RDC. Our data corroborate that CDC could effectively stymie the elevation of UCH-L1 and GFAP levels in the plasma. IF assay showed that the numbers of both UCH-L1-positive and GFAP-positive cells in the CDC group were decreased to varying degrees, in comparison with those in the RDC group. In addition, FJ-C staining confirmed the potent efficacy of CDC in alleviating cortical neuronal degeneration. These results comprehensively and cogently demonstrate that CDC manifested superior neuroprotective effects to RDC.

AICH induced by severe TBI, cerebral hemorrhage, and other CNS diseases pose a daunting challenge to the medical community, as the acutely increased intracranial pressure would displace brain tissue, facilitate the formation of brain herniation in certain severe cases, and thereby endanger the prognosis and the survival of the patients. The early phase management of AICH by applying decompressive craniectomy could enlarge the intracranial space for the brain tissue under hypertension to reduce intracranial pressure, facilitating the reconstruction of cerebral blood perfusion, and assuaging secondary brain injury [16]. However, the unfavorable complications caused by decompressive craniectomy, such as delayed hematoma, acute intraoperative brain swelling, and postoperative cerebral infarction, make it infeasible to reduce the incidence of vegetative state and the high disability rate of patients [17]. In an attempt to realize the gradual recovery of cerebral blood volume and alleviate ischemia-reperfusion injury, our team reported a novel surgical approach named CDC. The surgery features real-time monitoring of the changes of intracranial pressure (ICP) throughout the decompressive procedure of craniotomy in patients with acute cranial hypertension to lower ICP by various means and thereby contributing to the gradual and effective reperfusion of brain tissue [18]. The efficacy of CDC was demonstrated in a clinical trial of patients with severe TBI, as the patients reported improved 6-month prognosis, lower incidence of intraoperative acute brain swelling, and delayed intracranial hematoma than those who underwent RDC [9]. Despite the pronounced therapeutic effect of CDC in clinical practice, few studies have been conducted to evaluate its efficacy from the perspective of biomarkers and to explore the molecular mechanism of alleviating brain injury from oxidative injury and neuroinflammation.

The article "Controlled Decompression Alleviates Brain Injury via Attenuating Oxidative Damage and Neuroinflammation in Acute Intracranial Hypertension" was retracted in 2023. Reasons: signs of a paper mill; compromised peer review; unreliable results or conclusions.

MDA can be formed from arachidonic acid (AA), linoleic acid, and a-linolenic acid. As a commonly measured endpoint of reactive oxygen species- (ROS-) induced lipid peroxidation, MDA level correlates with the degree of ROS-induced damage [19]. Unlike MDA, AA is the only source of 8-iso-PGF2*α*, and measurement of 8-iso-PGF2*α* can offer a dependable path for quantitative measurement of oxidative stress status. In acute neurological diseases, such as TBI, 8-iso-PGF can be produced by astrocytes, which cause vasoconstriction and reduced posttraumatic cerebral blood flow [20]. Thus, we examined MDA and 8-iso-PGF2*α*, which are indicators of oxidative damage [21]. Meanwhile, the adverse effects of ROS are countered by the antioxidant enzymes SOD. SOD can convert superoxide radicals to H_2_O_2_, thus dampening the impacts of the radicals [22]. Oxidative stress is the result of ROS production exceeding the antioxidant buffer capacity, ensued by continuous accumulation of harmful products, which damages cellular macromolecules and is closely associated with aging, disease, and even death [23]. Our research suggested that MDA and 8-iso-PGF2*α* levels in plasma and cortex significantly increased and SOD activity decreased after AICH, and this trend can be ameliorated by CDC, rather than RDC. The plasma MDA level began to increase immediately after surgery and began to decrease 24 h later, while the plasma 8-iso-PGF2*α* level increased significantly at 6 h postoperatively and still showed a slow upward trend until 72 h in the rabbit AICH model. This result suggested that plasma MDA responded more quickly than 8-iso-PGF2*α*, while the elevation of 8-iso-PGF2*α* in plasma sustained longer after AICH.

The article "Controlled Decompression Alleviates Brain Injury via Attenuating Oxidative Damage and Neuroinflammation in Acute Intracranial Hypertension" was retracted in 2023. Reasons: signs of a paper mill; compromised peer review; unreliable results or conclusions.

Neuroinflammation is a double-edged sword that plays a complex role in different pathophysiological processes. It is generally believed that neural tissue can suppress infection through neuroinflammation and clear away damaged cell fragments and toxic metabolites, but the persistence of neuroinflammation is harmful to CNS cells [24]. An increasing body of evidence suggests that neuroinflammation induced by various pathophysiological processes such as oxidative stress plays a crucial role in the pathogenesis of acute CNS diseases, including brain injury [25, 26]. In the course of acute CNS diseases, microglia and astrocytes respond rapidly to external stimuli, so as to maintain CNS homeostasis. Liddelow et al. reported that activated microglia can not only affect neuronal connections but also induce neurotoxic astrocytes by secreting IL-1*α* and TNF when there is CNS injury. These newly formed astrocytes lose the ability to promote neuronal survival, outgrowth, and synaptogenesis and might be harmful to neurons [27]. Our study also showed that inflammatory cytokine expression is increased in the early stages of acute cranial hypertension, as is the expression of the astrocyte marker GFAP. In addition, we observed that CDC after AICH showed an inhibitory effect on the high expression of inflammatory cytokines, including TNF-*α*, IL-1*β*, IL-6, and IL-8. These results provide solid evidence substantiating the neuroprotective effect of CDC against acute inflammation in the rabbit brain.

Neuron-derived UCH-L1 and astrocyte-derived GFAP in tandem have been employed in the diagnosis of the severity of cranial brain injury in several clinical and animal studies [12, 28]. Evidence suggested that UCH-L1 could be detected in the plasma and cerebrospinal fluid as early as 2 hours after injury, and its level persisted until 24 hours in the chronic constriction injury (CCI) model of rat [29]. Zoltewicz et al. found that GFAP expression was significantly increased in the injured cortex on day 7 post-TBI, and the dramatically increased CSF level on day 1 postinjury was indicative of the severity of injury in a penetrating brain injury (PBI) model of rat [30]. Analogously, an increasing number of clinical trials have confirmed that increased UCH-L1 and GFAP expression post-TBI could be applied in the assessment of the severity of the injury and the clinical prognosis of TBI patients [31, 32].

The article "Controlled Decompression Alleviates Brain Injury via Attenuating Oxidative Damage and Neuroinflammation in Acute Intracranial Hypertension" was retracted in 2023. Reasons: signs of a paper mill; compromised peer review; unreliable results or conclusions.

In the current study, we constructed a rabbit model of AICH and examined the changing patterns of UCH-L1 and GFAP in plasma 2 days prior to operation and at 3, 6, 24, and 72 hours after the operation. Our data showed that plasma UCH-L1 peaked in the CDC group and RDC group at 3 h postsurgery, yet was not significantly different from that in the SH group 24 h later. Plasma GFAP levels in the CDC group and RDC group commenced soaring at 3 h postoperatively and remained significantly higher at 24 h postoperatively than that in the SH group. Such an aberrant increasing trend is generally consistent with previous studies [33]. The negligible amount of GFAP in the plasma of the SH group at all time points concurs with the finding of previous findings and could probably be attributed to the notion that the relatively large molecular weight of GFAP hinders its passage through the blood-brain barrier under normal physiological conditions [34]. In contrast, the expression of UCH-L1 in the plasma of all groups before surgery reveals that UCH-L1 is distributed in the plasma under physiological conditions; however, its source remains to be clarified [35, 36]. In the current experiment, we could not collect cerebrospinal fluid to analyze the kinetics and metabolism of UCH-L1 and GFAP in cerebrospinal fluid, owing to the restriction of experimental animals and techniques; hence, further studies are needed to verify the expression patterns of UCH-L1 and GFAP in the cerebrospinal fluid after CDC for the treatment of AICH in rabbits. Moreover, our animal model has certain limitations. ICP probes are implanted into the brain of the animal, and the ensuing damage cannot be dismissed. Our previous studies have suggested that CDC functions to alleviate ischemia-reperfusion injury. Although it was preliminarily confirmed in this study that CDC alleviates brain injury by alleviating oxidative damage and neuroinflammation, the molecular mechanism of the neuroprotective effect of CDC still needs to be explored.

To our knowledge, this is the first experimental study to verify the neuroprotective effect of CDC in the AICH model of rabbits by analyzing the levels of UCH-L1 and GFAP. As a new technique, the exploration into the exact molecular mechanism underlying the neuroprotective effect of CDC will contribute to its broader application in clinical practice. Our study demonstrates that CDC improves neurological function, lowers brain water content, and ameliorates neuronal degeneration, most probably via reducing oxidative stress injury and neuroinflammation.

The article "Controlled Decompression Alleviates Brain Injury via Attenuating Oxidative Damage and Neuroinflammation in Acute Intracranial Hypertension" was retracted in 2023. Reasons: signs of a paper mill; compromised peer review; unreliable results or conclusions.

## Figures and Tables

**Figure 1:** CDC attenuates brain damage following AICH. (a) Neurological function score in rabbits at 24 h postoperatively (*n* = 12). (b) Brain water content (%) (*n* = 12). (c) Typical images of FJ-C staining in rabbits at 3 h postoperatively (*n* = 6, scale bar = 50 *μ*m). Data are expressed as mean ± SD. ^∗^*P* < 0.05 vs. RDC; ^∗∗∗^*P* < 0.001 vs. RDC; ^###^*P* < 0.001 vs. SH.

**Figure 2:** The antioxidative effects of CDC. (a) MDA content in plasma. (b) 8-iso-PGF2*α* content in plasma. (c) SOD content in plasma. Expression of (d) MDA, (e) 8-iso-PGF2*α*, and (f) SOD in the cortex of rabbit at 24 h after operation. Data are expressed as mean ± SD, *n* = 6. ^∗∗^*P* < 0.01 vs. RDC; ^∗∗∗^*P* < 0.001 vs. RDC; ^#^*P* < 0.05 vs. SH; ^##^*P* < 0.01 vs. SH; ^###^*P* < 0.001 vs. SH.

**Figure 3:** The anti-inflammatory effects of CDC. The mRNA levels of TNF-*α* (a), IL-1*β* (b), IL-6 (c), and IL-8 (d) in the cerebral cortex of rabbits at 24 h postoperatively. Expression of (e) TNF-*α*, (f) IL-1*β*, (g) IL-6, and (h) IL-8 in the plasma at 24 h after operation. Data are expressed as mean ± SD, *n* = 6. ^∗^*P* < 0.05 vs. rapid group; ^∗∗^*P* < 0.01 vs. RDC; ^∗∗∗^*P* < 0.001 vs. RDC; ^#^*P* < 0.05 vs. SH; ^##^*P* < 0.01 vs. SH; ^###^*P* < 0.001 vs. SH.

**Figure 4:** Immunofluorescence (IF) staining of UCH-L1 and GFAP in cortex tissues. (a) The left panel shows IF staining of UCH-L1 in rabbit cortex 3 h after surgery; the right panel displays the percentage of UCH-L1-positive cells. (b) The left panel shows IF staining of GFAP in rabbit cortex 3 h after surgery; the right panel exhibits the percentage of GFAP-positive cells. Scale bar = 50 *μ*m. Data are expressed as mean ± SD, *n* = 6. ^∗∗^*P* < 0.01 vs. rapid group; ^∗∗∗^*P* < 0.001 vs. rapid group; ^###^*P* < 0.001 vs. sham group.

**Figure 5:** RT-qPCR was performed to analyze mRNA levels of UCH-L1 (a) and GFAP (b) in the cortex of rabbits. Data are expressed as mean ± SD, *n* = 6. ^∗^*P* < 0.05 vs. RDC; ^∗∗^*P* < 0.01 vs. RDC; ^∗∗∗^*P* < 0.001 vs. RDC; ^#^*P* < 0.05 vs. SH; ^###^*P* < 0.001 vs. SH. ns: not significant.

**Figure 6:** The expression levels of UCH-L1 and GFAP were measured by performing ELISA and Western blotting. (a) The serum levels of UCH-L1 at each time point in three groups of rabbits. (b) The serum levels of GFAP at each time point in three groups of rabbits. (c) Western blotting assay of UCH-L1 and GFAP protein expressions in cortex at 3 h postoperatively. The intensities of interesting signals were compared. Data are expressed as mean ± SD, *n* = 6. ^∗^*P* < 0.05 vs. RDC; ^∗∗∗^*P* < 0.001 vs. RDC; ^#^*P* < 0.05 vs. SH; ^###^*P* < 0.001 vs. SH.

The article "Controlled Decompression Alleviates Brain Injury via Attenuating Oxidative Damage and Neuroinflammation in Acute Intracranial Hypertension" was retracted in 2023. Reasons: signs of a paper mill; compromised peer review; unreliable results or conclusions.

## Data Availability

The data used to support this study are available from the corresponding authors upon request.
